RETRACTED

# Analysis of the Influence of High-Dose rhGH Therapy on Serum Vitamin D and IGF-1 Levels in School-Age Children with Idiopathic Short Stature

**DOI:** 10.1155/2021/5776487

**Published:** 2021-10-26

**Authors:** Juan Li, Xuehui Zhang, Shuyong Xie, Shuangshuang Feng, Min Niu

**Affiliations:** Endocrine Department, Anhui Fuyang People's Hospital, Fuyang, Anhui 236000, China

## Abstract

**Objective:**

To discuss the influence of high-dose recombinant human growth hormone (rhGH) therapy on serum vitamin D and insulin-like growth factor-1 (IGF-1) levels in school-age children with idiopathic short stature (ISS).

**Method:**

A total of 103 school-age children with ISS were selected from June 2016 to June 2020 in our hospital. The enrolled cases were divided into the low-dose group (*n* = 59) and high-dose group (*n* = 44) according to the treatment dose of rhGH. After the treatment, the height (Ht), height standard deviation score (Ht SDS), growth velocity (GV), and other indicators were recorded. The serum 25-hydroxy vitamin D [25-(OH)D] and IGF-1 levels of the two groups were tested, and the occurrence of adverse reactions was recorded.

**Results:**

After treatment, the high-dose group outperformed the low-dose group in various growth effect indicators such as Ht, Ht SDS, and GV (*P* < 0.05). After treatment, the serum 25-(OH)D of children with ISS in the two groups increased significantly, but there was no significant difference between the two groups (*P* > 0.05). After treatment, the serum IGF-1 of children with ISS in the two groups increased significantly, but there was no significant difference between the two groups (*P* > 0.05). For children with ISS, adverse reactions induced by rhGH therapy were very rare. There was no significant difference in the incidence of adverse reactions induced by different doses of rhGH in the treatment of ISS (*P* > 0.05).

**Conclusion:**

rhGH has definite efficacy in the treatment of ISS children, for it can significantly increase the annual growth rate of ISS children in a dose-dependent manner. High-dose rhGH for ISS has a better therapeutic effect. At the same time, regardless of the dose level of rhGH, serum 25-(OH)D and IGF-1 levels in children with ISS were increased, with less adverse reactions and higher safety.

## 1. Introduction

Childhood short stature is a growth and development disorder with a high prevalence. According to statistics, the research results released by the WHO in 2000 showed that the prevalence of short stature had a great correlation with the degree of national economic development. In some economically backward regions, the prevalence of short stature was as high as 32.5% [1]. In the United States, there are up to 5 children with short stature for every 100 infants [2]. Short stature is associated with a variety of factors, including growth hormone deficiency, growth hormone neurosecretory disorder, intrauterine growth retardation, idiopathic short stature, hypothyroidism, and nutritional deficiency. Among them, idiopathic short stature (ISS) is the most common type of short stature, accounting for 60%–80% of children with short stature [3]. ISS refers to that the height of the child is lower than that of the child of the same age and gender by two standard deviations, the general height and weight at birth are normal, and there is no evidence to support systemic, endocrine, nutritional, and chromosomal abnormalities. ISS is a disease of symmetrical short stature, and there is no clear cause in clinical practice [4]. School-age children's emotions are relatively fragile. If children have short stature, it is easy to cause children's life, behavior, and psychological disorders. In interpersonal communication, children are often frustrated for various reasons, which leads to children lagging behind their peers in social interaction, thus leading to different degrees of psychological problems [5]. Therefore, effective treatment for school-age children with ISS is urgently needed.

RETRACTED

Recombinant human growth hormone (rhGH) is currently the most commonly used and effective drug for the clinical treatment of ISS. rhGH can stimulate the liver and other organs to produce insulin-like growth factor-1(IGF-1), act on the chondrocytes in the epiphyseal plate, facilitate the synthesis of collagen and mucopolysaccharide sulfate, and promote and affect the synthesis and metabolism of protein, thereby playing a role in promoting bone growth [6, 7]. However, the optimal dose of rhGH has always been a hot topic in the treatment of children with ISS.

Studies have shown that more than 95% of active vitamin D in serum is 25-hydroxy vitamin D [25-(OH)D], and serum 25-(OH)D is the most abundant vitamin D of multiple vitamin D metabolites in serum, followed by 1,25-(OH)_2_D. Although serum 1,25-(OH)_2_D has the highest biological activity, the half-life of this indicator is short and it is difficult to be quantitatively detected. 25-(OH)D has long been existed in the body and good stability, so it is currently considered to be an important indicator reflecting the vitamin D level of the body. This indicator can regulate the metabolism of calcium and phosphorus in the human body and promote calcium absorption and reabsorption, as well as bone deposition, and has a positive effect on the maintenance of bone health [8]. IGF-1, a single-chain polypeptide, is mainly produced by the liver, skeletal muscle, and many other tissues in response to growth hormone (GH) stimulation. It promotes the growth and differentiation of bones and tissues, as well as the production of muscle mass, thus exerting an important regulatory effect on the body's growth. IGF-1 is closely related to the GH level. The synthesis and secretion of IGF-1 are regulated by the GH level, while the IGF-1 level can form negative feedback to regulate the secretion of growth hormone by the pituitary gland. At the same time, IGF-1 also plays a key role in the nongrowth activities of glucose and fat metabolism and metabolic syndrome [9].

RETRACTED

In China, pediatric clinical practice recommends that the therapeutic dose of rhGH is 0.1–0.2 IU/kg per day. Because of its certain degree of growth hormone resistance, it is recommended that the therapeutic dose of rhGH is higher than that for other diseases. Therefore, in this study, 0.15 IU/kg rhGH was used as the boundary group, and 103 school-age children with ISS were selected for investigation. The therapeutic effects of different doses of rhGH and the effects on serum 25-(OH)D and IGF-1 levels were observed, in order to guide clinical treatment and make the lifetime height of children with ISS reach the normal age-appropriate height.

## 2. Methods

### 2.1. General Information

A total of 103 school-age children with ISS were selected from June 2016 to June 2020 in our hospital. There were 57 males and 46 females, aged from 6 to 13 years old, with the average age of (9.25 ± 2.37) years old.

Diagnostic criteria for ISS were defined as follows: (1) height was less than 2 standard deviations of the mean or lower than the 3rd percentile of the mean, compared with children of the same age, gender, and race; (2) the body length and weight at birth develop normally, the limbs develop well, and there was no intrauterine growth retardation; (3) there was no obvious chronic organic disease, such as heart, lung, liver and kidney, endocrine, and metabolic abnormalities and bone development disorders; (4) no chromosome abnormality; (5) eating normally, without significant or severe emotional disorders; (6) the growth and development were close to or later than those of the normal population; and (7) the growth hormone peaks in the above two growth hormone challenge tests exceeded 10 ug/L and the normal IGF-1 concentration in blood.

Inclusion criteria were defined as follows: met the diagnostic criteria for ISS; slow growth; complete clinical data; and families were informed of the content of the study.

Exclusion criteria were defined as follows: malnutrition; endocrine genetic metabolic diseases; growth retardation caused by various chronic diseases; those who were being investigated or treated in other clinical studies; children with irregular medication and regular follow-up; history of rhGH therapy; severe liver and kidney dysfunction; and combined with Turner syndrome; combined with precocious puberty.

RETRACTED

### 2.2. Research Methods

#### 2.2.1. Treatment Plan and Grouping

The enrolled cases were divided into two groups according to the treatment dose of rhGH: low-dose group (*n* = 59), with the treatment dose ranging from 0.10 to 0.15 IU/kg per day, and high-dose group (*n* = 44), with the treatment dose ranging from 0.16 to 0.20 IU/kg per day. The dose range was based on the guidelines for the diagnosis and treatment of short stature children. All the children received subcutaneous injection of rhGH 1 h before bedtime every night from the lateral thigh to the navel. The injection site was changed every time, and the treatment course was 6–24 months. At the same time, during the treatment, doctors need to inform the parents of patients that they need to reasonably arrange the diet, sleep, and exercise conditions of children, guided children to carry out specific sports in an appropriate amount, and eat healthy and scientific to ensure adequate sleep. Height (Ht), weight, body mass index (BMI) = weight/height (Ht)^2^, and general physical examination were reviewed every 3 months, and the changes of fasting blood glucose, serum vitamin D, and IGF-1 levels were monitored.

#### 2.2.2. Assessment Indicators

After the treatment, the Ht, height standard deviation score (Ht SDS), growth velocity (GV), and other indicators were recorded to evaluate the effect of the treatment on children receiving rhGH treatment. In the past, the standard for Ht measurement was based on “the National Standards for Physical Fitness and Health for Students”. Before the measurement, the Ht and weight measuring instrument was calibrated and reset to zero, and the shoes and socks were removed. During the measurement, the child was asked to raise his head and chest, the upper limbs were in a natural drooping state, the legs and heels were brought together, the eyes were straight ahead, the posture was standing upright, and the measurement was repeated 3 times, and the average value was taken. Ht SDS = (actual height of children − median height of normal children of the same sex and age)/standard deviation of height of normal children of the same sex and age. The height standard was based on the data of the children's physical development survey in 9 provinces/cities in China in 2005. GV = (height at posttreatment follow-up − height at initiation of treatment)/time interval (months) × 12.

RETRACTED

Fasting venous blood was collected at 4 mL in the morning and centrifuged at 2500 r/min for 5 min before treatment and 6, 12, and 24 months after treatment. The supernatant was collected, and serum was separated and stored in a −80°C refrigerator. Chemiluminescent enzyme immunoassay was used as the detection method: serum 25-(OH)D was detected using ELISA immunoassay, and serum IGF-1 concentration was determined using the chemiluminescent method. The specific operations were performed strictly following the instructions.

During the treatment, we observed whether the children had adverse reactions, including elevated fasting glucose, edema, red and swollen injection site, rash, arthrodynia, and other symptoms.

### 2.3. Statistical Methods

SPSS 22.0 statistical software was used for data processing, and the enumeration data were expressed as rate (%). The *χ*^2^ test was used for comparison. Measurement data were expressed as ($\bar{x}$ ± *s*), and comparison was performed using the *t*-test or variance test. *P* < 0.05 indicated that the difference was statistically significant.

## 3. Results

### 3.1. Comparison of Baseline Data between the Two Groups before Treatment

Before treatment, the baseline data such as age, gender, BMI, fasting blood glucose, Ht, Ht SDS, and GV of the two groups were not statistically significant (*P* > 0.05) (see Table 1).

### 3.2. Comparison of the Effects of Different Doses of rhGH in the Treatment of ISS

After treatment, the high-dose group outperformed the low-dose group in various growth effect indicators such as Ht, Ht SDS, and GV (*P* < 0.05) (see Table 2).

### 3.3. Changes of Serum 25-(OH)D before and after Treatment of ISS with Different Doses of rhGH

After treatment, the serum 25-(OH)D of children with ISS in the two groups increased significantly, but there was no significant difference between the two groups (*P* > 0.05) (see Table 3).

### 3.4. Changes of Serum IGF-1 before and after Treatment of ISS with Different Doses of rhGH

After treatment, the serum IGF-1 of children with ISS in the two groups increased significantly, but there was no significant difference between the two groups (*P* > 0.05) (see Table 4).

### 3.5. Adverse Reactions of Different Doses of rhGH in the Treatment of ISS

For children with ISS, adverse reactions induced by rhGH therapy were very rare. There was no significant difference in the incidence of adverse reactions induced by different doses of rhGH in the treatment of ISS (*P* > 0.05) (see Table 5).

## 4. Discussion

ISS is a group of short stature syndrome with unclear cause. The causes of ISS are various and complex, and the common causes include GH receptor gene mutation, short homeobox gene deletion, GH secretion dysfunction, and structural abnormalities [10]. ISS not only affects children's height but also easily leads to abnormal bone development, nervous system dysfunction, and the increased incidence of chronic cardiopulmonary diseases and will have a great impact on children's life quality in the future [11]. Therefore, it is clinically necessary to implement a scientific treatment plan for children with ISS.

RETRACTED

Application of rhGH before complete epiphysis closure is the most important and effective treatment for ISS. Human GH is a peptide hormone secreted by GH-secreting cells containing eosinophilic granules in the anterior pituitary gland and is the most important hormone for promoting growth after human birth. GH has a wide range of physiological effects. It can promote the growth and development of tissues and regulate the metabolism of sugar, protein, and fat in the body. For GH to promote growth, it must first bind to cell surface-specific receptors to form ligand-receptor complexes, which then mediate and trigger a series of biochemical reactions by the receptors to finally start the transcription of GH target genes and produce active factors to exert biological effects [12, 13]. rhGH is produced and obtained by recombinant DNA technology, and its chemical structure is identical to that of GH secreted by the pituitary gland. At present, many studies have shown that, although children with ISS have no GH deficiency, the use of rhGH therapy for ISS children can help accelerate the growth process of children [14]. In 2003, the US Food and Drug Administration approved the use of rhGH in the treatment of children with ISS. The safe and effective application of rhGH has been widely recognized in clinical practice [15]. However, the dose selection of rhGH in the treatment of children with ISS has always been a key issue of clinical concern.

Hokken-Koelega's team [16] performed rhGH treatment on children with small for gestational age (SGA) dwarfism and divided the children into a low-dose group (0.033 mg/kg per day, equivalent to 0.1 IU/kg per day) and a high-dose group (0.067 mg/kg per day, equivalent to 0.2 IU/kg per day). The height growth of the two groups reached two standard deviations after 5.5 and 2.5 years of treatment. The results suggested that the high-dose rhGH group could achieve significant catch-up growth effect earlier than the low-dose rhGH group. There are many etiologies of ISS, and the causes are complex and diverse. Therefore, there are differences in the effect and sensitivity of rhGH treatment for children with ISS. The increase in stimulation to growth hormone receptor can be achieved clinically by increasing that dose of rhGH, which in turn increases the receptor's sensitivity to rhGH. The expression activity of growth hormone receptor was positively correlated with the increase in rhGH concentration, and the gene sites were polymorphic, so the amount of rhGH was one of the important factors affecting the therapeutic effect of ISS. The results of this study showed that after the treatment, the growth effect indicators such as Ht, Ht SDS, and GV in the high-dose group were superior to those in the low-dose group. The results can reveal that rhGH has a definite therapeutic effect on ISS children and can significantly increase the annual growth rate of ISS children. In addition, the curative effect is in a dose-dependent manner, and high-dose rhGH for ISS has a better therapeutic effect.

RETRACTED

We found that after treatment, the serum 25-(OH)D and IGF-1 of children with ISS in the two groups were increased significantly, but there was no significant difference between the two groups, indicating that regardless of the dose level of rhGH, the serum 25-(OH)D and IGF-1 levels of children with ISS were increased, and the growth effect was promoted. Ameri's team [17] found a high risk of vitamin D deficiency in children with GH deficiency but improved vitamin D deficiency after 12 months of rhGH treatment. Vitamin D plays an important regulatory role in the absorption of calcium and phosphorus in the human body, which is conducive to promoting the normal mineralization of bones. School-age children are vulnerable to vitamin D deficiency. Serum 25-(OH)D is an active product of the metabolism of vitamin D by the liver, and insufficient synthesis of 25-(OH)D will affect the absorption and metabolism of calcium and phosphorus by the body, reducing the concentration of calcium and phosphorus in serum, and then the mineralization function of osteoblasts is hindered in the synthesis of bone matrix and collagen fiber, which in turn affects the height growth of children [18]. Our study suggested that rhGH might stimulate the synthesis of serum 25-(OH)D in children with ISS and there was no rhGH dose-dependent level of 25-(OH)D. However, the specific mechanism of this conclusion is still unclear, and further research is needed. We suggested that the possible mechanism is that vitamin D 25-hydroxylation occurs in liver mitochondria and microsomes and cytochrome P-450 enzyme is involved in this process. GH can enhance the P-450 activity of liver mitochondria through direct action or indirect action of IGF-1, thereby inducing the activation of vitamin D; GH may enhance renal 1*α*-hydroxylase activity by IGF-1, thereby inducing vitamin D activation and elevated serum 25-(OH)D levels. GH treatment accelerates the growth of children with ISS and may result in relative calcium and phosphorus deficiency, while low calcium and phosphate levels increase renal 1*α*-hydroxylase activity and thus serum 25-(OH)D levels. In addition, human growth is an extremely complex biological process, and the hypothalamic-GH-IGF-1 axis is the main endocrine system that regulates human growth. Under normal circumstances, GH stimulates the production of IGF-1 as an auxin medium to play a role in promoting bone growth, regulating body metabolism, and promoting the synthesis of protein. Compared with normal children, children with ISS have lower serum IGF-1 content, and the most critical growth and development regulator in childhood is IGF-1 [19]. After the treatment of children with ISS with rhGH, we found that it can promote the production of IGF-1 in the liver, significantly increase the release of IGF-1, and promote cell growth and differentiation, thereby improving bone growth in children.

RETRACTED

In addition, adverse reactions to the rhGH regimen in children with ISS were rare in this study. One case of rash appeared in the low-dose group, and the symptoms of the child resolved spontaneously without special treatment. One patient in the high-dose group had elevated fasting blood glucose, which did not reach the level of diabetes in children. Without special treatment, the blood glucose of the child dropped to the normal range. One case in the high-dose group developed early lower limb edema, and all the children's symptoms resolved spontaneously without special treatment. One child in the high-dose group had knee pain, which might be growth pain, and the pain in the child was relieved after calcium supplementation. Clinically, rhGH treatment programs also have other adverse effects, including hypothyroidism, benign intracranial hypertension, scoliosis, myalgia, arthralgia, slippage of the femoral head, enlarged hands and feet, etc. In this study, none of the children with ISS had the above-mentioned adverse reactions. We found that rhGH has high safety in the treatment of ISS in children, with less adverse reactions.

## 5. Conclusion

Recombinant human growth hormonehas definite efficacy in the treatment of ISS children, for it can significantly increase the annual growth rate of ISS children in a dose-dependent manner. High-dose rhGH for ISS has a better therapeutic effect. At the same time, regardless of the dose level of rhGH, serum 25-(OH)D and IGF-1 levels in children with ISS were increased, with less adverse reactions and higher safety. For children with slow-growing ISS, rhGH should be used early in clinical practice. If the family economic conditions of the children allow it and the expectation of final adult height is high, high dose of rhGH can be used for treatment in the first year as far as possible within a safe range, and then different degrees of individual adjustment can be made according to the growth rate of children in the first year to achieve the best effective treatment effect.

RETRACTED

## Figures and Tables

**Table 1:** Comparison of baseline data between the two groups before treatment (*n*, %, $\bar{x}$ ± *s*).

Group	Number of cases	Age (years)	Gender		BMI (kg/m^2^)
			Male	Female	
Low-dose group	59	9.34 ± 2.08	30(50.85%)	29(49.15%)	14.65 ± 1.53
High-dose group	44	9.13 ± 2.42	27(61.36%)	17(38.64%)	14.72 ± 1.57
*t*/*χ*^2^ value		0.472	1.128	0.227	
*P* value		0.637	0.288	0.821	
Group	Number of cases	Fasting blood glucose (mmol/L)	Ht (cm)	Ht SDS	GV (cm/y)
Low-dose group	59	4.79 ± 0.48	120.96 ± 16.33	−2.81 ± 0.94	4.13 ± 0.40
High-dose group	44	4.72 ± 0.50	121.45 ± 15.08	−2.86 ± 0.99	4.07 ± 0.45
*t* value		0.719	0.198	0.261	0.713
*P* value		0.473	0.843	0.794	0.477

**Table 2:** Comparison of the effects of different doses of rhGH in the treatment of ISS (*n*, $\bar{x}$ ± *s*).

Group	Number of cases	Ht (cm)	Ht SDS	GV (cm/y)
Low-dose group	59	140.37 ± 18.02	−2.12 ± 0.90	7.28 ± 1.25
High-dose group	44	147.95 ± 19.63	−1.24 ± 0.86	8.03 ± 1.44
*t* value		2.032	5.002	2.822
*P* value		0.044	≤0.001	0.006

**Table 3:** Changes of serum 25-(OH)D before and after treatment of ISS with different doses of rhGH (*n*, $\bar{x}$ ± *s*, ng/mL).

Group	Number of cases	Before treatment	6 months after treatment	12 months after treatment	24 months after treatment
Low-dose group	59	36.41 ± 9.80	39.50 ± 11.65^*∗*^	46.12 ± 14.79^*∗*^	52.06 ± 16.51^*∗*^
High-dose group	44	34.67 ± 10.19	40.79 ± 12.33^*∗*^	48.26 ± 15.82^*∗*^	52.13 ± 16.30^*∗*^
*t* value		0.876	0.542	0.705	0.021
*P* value		0.382	0.588	0.482	0.983

*Note.* Compared with that before treatment, ^*∗*^*P* < 0.05.

**Table 4:** Changes of serum IGF-1 before and after treatment of ISS with different doses of rhGH (*n*, $\bar{x}$ ± *s*, ng/mL).

Group	Number of cases	Before treatment	6 months after treatment	12 months after treatment	24 months after treatment
Low-dose group	59	129.85 ± 81.64	262.67 ± 102.55^*∗*^	384.40 ± 98.36^*∗*^	447.53 ± 77.65^*∗*^
High-dose group	44	131.09 ± 80.31	295.43 ± 104.68^*∗*^	357.15 ± 80.54^*∗*^	461.62 ± 73.21^*∗*^
*t* value		0.076	1.589	1.500	0.933
*P* value		0.938	0.115	0.136	0.352

*Note.* Compared with that before treatment, ^*∗*^*P* < 0.05.

**Table 5:** Adverse reactions of different doses of rhGH in the treatment of ISS (*n*, %).

Group	Number of cases	Elevated fasting glucose	Edema	Red and swollen injection site	Rash	Arthrodynia	Total incidence
Low-dose group	59	0	0	0	1	0	1(1.69%)
High-dose group	44	1	1	0	0	1	3(6.82%)
*χ* ^2^ value							1.772
*P* value							0.183

RETRACTED

## Data Availability

The data used and/or analyzed during the current study are available from the corresponding author upon request.
